The article "Application of Realistic 3D Model in Building Prefabricated Nanomaterial Structure" was retracted in 2023. Reasons: signs of a paper mill; suspected computer-generated content; unreliable results or conclusions; concerns about the data.

# Application of Realistic 3D Model in Building Prefabricated Nanomaterial Structure

**DOI:** 10.1155/2022/1726948

**Published:** 2022-08-04

**Authors:** Sihui Li

**Affiliations:** Yellow River Conservancy Technical Institute, Kaifeng 475003, Henan, China

## Abstract

In order to solve the problem of 3D modeling in building assembly, an application of a 3D model based on the real scene in the building assembly structure is proposed. This method, based on the current BIM technology in nanomaterial design research, analyzes the problems existing in the traditional assembly structure design scheme and analyzes the feasibility of BIM technology in the forward design of assembly buildings from the perspective of theory and practical application. The experimental results show that the urban building model established by the 3D model has high precision and a good real-scene effect. The accuracy of the building model meets the requirements of 1 : 1000 mapping, has measurable accuracy, and elevation accuracy is better than 30 cm. The 3D model promotes the development of informatization.

## 1. Introduction

The construction industry is an important support for China's economic development, which is closely related to the economic development of the whole country and related to people's living standards. With the Chinese people's living standards basically reaching a well-off level in the new century, in order to achieve the goal of building a moderately prosperous society in all respects, demands are put forward in economic construction and the improvement of people's living standards. Traditional construction methods have been far from meeting people's demand for high-quality construction products; At the same time, in the aspect of sustainable development and ecological environment construction, the state emphasizes the continuous enhancement of the ability to achieve sustainable development and the improvement of the efficiency of resource reuse. In the construction industry, in order to promote the continuous development of society, the construction method of prefabricated buildings has changed the traditional extensive construction method. Nanomaterials have become the focus of national development because of their advantages in saving resources and energy, reducing construction pollution, improving production efficiency and safety, etc., which conform to the development of The Times. With the development of intelligent equipment such as computer communication, information technology has been combined in the process of architectural design, production, and construction. The development of information technology has brought a new development direction to the cost of prefabricated buildings with high cost.

The article "Application of Realistic 3D Model in Building Prefabricated Nanomaterial Structure" was retracted in 2023. Reasons: signs of a paper mill; suspected computer-generated content; unreliable results or conclusions; concerns about the data.

## 2. Literature Review

Dubrovsky et al. say that BIM is a three-dimensional digital technology applied to the whole life cycle of buildings, creating and collecting building information and establishing coordinated information models as the basis for project decisions and resources to share Information [1]. Oqielat and others say BIM is not only a modeling tool but also an idea and approach throughout the entire life cycle of a building [2]. Mcgowan et al. said that the implementation of BIM technology is absolutely not dependent on a single software, but in the process of architectural design, construction, and operation and maintenance, all parties cooperate [3]. According to Zhao et al., compared with the 2D mapping mode with CAD software as the core, BIM technology has attracted much attention because of its visualization, parameterization, coordination, simulation, and graphability [4]. Lan et al. say that BIM technology has five characteristics: visualization: what you see is what you get. It is no longer a 2D plane drawing mode with CAD as the core, but a 3D model is provided for designers to help them analyze architecture deeply and select the optimal scheme. The communication and decision-making involved in the whole life-cycle process of the project (design, construction, and operation) are carried out under visualization [5]. Sarker et al. say that BIM technology provides not only a simple 3D model, but also a database containing a large amount of information and components combining a large amount of information into the whole building information model [6]. Zhang et al. said that in the design process, due to the lack of communication and coordination among various professional designers, the design will be unreasonable, causing great inconvenience to the later construction and operation and maintenance [7]. Jiang et al. say that BIM technology can closely correlate data, and the linkage between data is real-time and consistent [8]. Any changes to model data can be reflected in real time where they are associated and provide optimal solutions for designers. Lyu et al. said that various simulations could be carried out through the 3D data model designed, such as the analysis of net height, simulation of an emergency evacuation, simulation of energy saving, etc., so that problems could be found and solved early by simulation before the delivery of drawings [9]. Woniak et al. said that BIM-related design software can produce three-dimensional drawings, which can reduce human errors in the process of construction and operation and maintenance [10]. The first significant change in the field of engineering design is the emergence of CAD technology, designers completed the transformation from manual drawing to computer drawing. The emergence of BIM technology is an important change in the whole construction industry. The emergence of BIM technology has changed the situation of working alone in all fields of the construction industry. As an important carrier, the BIM model plays an irreplaceable role in EPC mode assembly building FM (Equipment management) CIM (Urban Building Information Model) In the Internet of Things (see Figure 1).

The article "Application of Realistic 3D Model in Building Prefabricated Nanomaterial Structure" was retracted in 2023. Reasons: signs of a paper mill; suspected computer-generated content; unreliable results or conclusions; concerns about the data.

## 3. Method

The 3D model of urban real scene is to restore the physical world with a high-precision model and real texture, so the way of obtaining texture is particularly important [11]. Manual shooting with the digital camera is not only inefficient, but also a single visual angle. The traditional aerial and aerospace photogrammetry technique is mainly used to measure the top of topographic features, but the description of the sides and geometric structure of features is very limited. As a new and high technology developed internationally in recent years, oblique photogrammetric technology can obtain images from different angles of ground objects and provide rich textures for the construction of the city three-dimensional model, which can solve the above problems well [12, 13]. Oblique photogrammetry, as a multi-angle photogrammetry technology, carries multiple sensors on the flight platform and shoots images from five different angles, such as vertical tilt, to obtain more complete and accurate information of ground objects [14]. The technology cannot only obtain orthophoto image of the photographed area, but also obtain the oblique image of the photographed area, record the location information of the shooting point, and realize the spatial positioning of the image through the late data processing. Traditional photogrammetry can only take images from vertical angles, but tilt photogrammetry overcomes this shortcoming and can take images from multiple angles. Because the tilted image contains complete geographical information, it can measure the height, length, and area of ground objects on the image [15]. In 3D modeling, it can provide rich ground object texture for 3D model and reduce the cost of modeling, as shown in Figure 2.

Inertial Navigation System (INS) is also called Inertial Measurement System (IM S). It consists of Inertial Measurement Unit (IMU) and a navigation computer. It is a navigation system that uses a high-precision gyroscope and accelerometer to measure the acceleration of the moving carrier, and then calculates the acceleration, attitude, and heading parameters of the moving carrier by computer [16]. INS is made up of an Inertial Measurement Unit (IMU) and a navigation computer and an IMU has three single-axis accelerometers and three single-axis gyroscopes. The accelerometer monitors the acceleration signal of the independent three axes of the object in the carrier coordinate system, and the gyro monitors the angular velocity signal of the carrier relative to the navigation coordinate system. An inertial navigation system, based on the law of inertial mechanics, calculates the acceleration of the moving carrier in the inertial coordinate system, integrates it into the inertial navigation system, and obtains the attitude information such as the speed yaw Angle of the moving carrier. However, the inertial navigation system has a fixed drift rate, which will produce deviation when the object moves. Therefore, it is necessary to use the instantaneous position information provided by GNSS to provide INS to eliminate the accumulated errors of the system. Second, INS needs GNSS to provide initial position and attitude parameters for acceleration conversion and integration calculation. Finally, due to the influence of the sampling rate of the satellite receiver, the instantaneous position information of the reference center of laser pulse transmission can only be provided by INS integral operation. In summary, the GNSS/INS combined position and attitude measurement system can greatly improve the accuracy of position and attitude parameters and overcome the error accumulation of INS. In the process of the tilted image obtained by the tilted photogrammetry technology, the principle of the space rear intersection and collinear condition of the traditional photogrammetry technology of the single image is mainly used, and the collinear condition equation is used to solve the external orientation elements of each single image, so as to solve and restore the spatial geographic location information of the tilted image. The basic principle of single space rear rendezvous is a method to obtain the external orientation elements of the image according to the ground coordinates (or ground photographic coordinates) of a certain number of control points in the shooting area and the corresponding image pixel coordinates. The collinearity condition equation is a mathematical expression expressing that the object point, the image point, and the photography center (i.e., the lens center of the image) are in a straight line, and its definition is shown in Figure 3.

The article "Application of Realistic 3D Model in Building Prefabricated Nanomaterial Structure" was retracted in 2023. Reasons: signs of a paper mill; suspected computer-generated content; unreliable results or conclusions; concerns about the data.

The calculation formula is shown in the formula below:

(1) $$\begin{array}{c} \left\{\begin{array}{c} X=-f\frac{a_{1}\left(X-X_{s}\right)+b_{1}\left(Y-Y_{s}\right)+c_{1}\left(Z-Z_{s}\right)}{a_{3}\left(X-X_{s}\right)+b_{3}\left(Y-Y_{s}\right)+c_{3}\left(Z-Z_{s}\right)}\\ Y=-f\frac{a_{2}\left(X-X_{s}\right)+b_{2}\left(Y-Y_{s}\right)+c_{2}\left(Z-Z_{s}\right)}{a_{3}\left(X-X_{s}\right)+b_{3}\left(Y-Y_{s}\right)+c_{3}\left(Z-Z_{s}\right)} \end{array}\right.. \end{array}$$

In the equation, *X* and *Y* are the coordinate value of image pixels, *f* is the focal length of the camera, and *X*, *Y*, and *Z* are the control point of the same name on the ground corresponding to the coordinate point of relative image pixels; *X*s, *Y*s, *Z*s are the video location line element for the camera when shooting video, *a*, *b*, *c*, their coefficients represent the angular elements of the picture. It is known from the collinear equation that the coefficient of the outer square element of the collinear equation requires at least three known ground control point pairs and pixel point pairs that are not on a straight line. Incline photogrammetry technology integrates dynamic GNSS positioning system inertial navigation system incline photogrammetry system to obtain multi-angle images of ground objects and provide rich and real textures for 3D modeling of urban real scenes [17]. Because the coordinate system is not parallel or the origin of the three coordinates is inconsistent, the position and attitude of POS can be naturalized to the center of the vertical camera through system checking and naturalization, and the external orientation elements of the vertical image can be obtained according to the POS data. Through the relative relationship between the tilted camera and the vertical camera, the external orientation elements of the tilted image are calculated, and then the tilted image of the vertical image is adjusted by the whole beam method to obtain the accurate external orientation elements of the image. It includes two steps: the calculation of relative position between cameras; Swdc-5 tilting camera can calculate the external orientation elements of each camera by using the pictures taken by the camera in the inspection field according to the space rear intersection, and then calculate the relative relationship between the tilting camera and the downward-looking camera according to the calculated line elements and relative Angle elements. Set the four tilted cameras as *A*, *B*, *C*, and *D*, and the downward-looking camera as *E*, where, the external azimuth element of camera B is (*X*_*B*_, *Y*_*B*_, *Z*_*B*_, *ϕ*_*B*_, *ω*_*B*_, *k*_*B*_), and the external azimuth element of camera *E* is (*X*_*B*_, *Y*_*B*_, *Z*_*B*_, *ϕ*_*B*_, *ω*_*B*_, *k*_*B*_), then the rotation matrix *R*_*E*_^*B*^ of camera B relative to camera *E* can be calculated as shown in the formula below:

(2) $$\begin{array}{c} R_{B}=R_{E}R_{E}^{B}\\ R_{E}^{B}=R_{B}R_{E}^{-1}. \end{array}$$

R_B_ and R_E_ are rotation matrices composed of corresponding Angle elements, and the relative line elements between cameras are shown in formula (3) in the object-square space coordinate system:

(3) $$\begin{array}{c} \left(\begin{array}{c} X_{BE}\\ Y_{BE}\\ Z_{BE} \end{array}\right)=\left(\begin{array}{c} X_{B}\\ Y_{B}\\ Z_{B} \end{array}\right)-\left(\begin{array}{c} X_{E}\\ Y_{E}\\ Z_{E} \end{array}\right). \end{array}$$

In the image space coordinate system, the relative position of camera *B* relative to camera *E* is shown in the formula below:

(4) $$\begin{array}{c} \left(\begin{array}{c} X_{BE}^{\prime }\\ Y_{BE}^{\prime }\\ Z_{BE}^{\prime } \end{array}\right)=R_{E}^{-1}\left(\begin{array}{c} X_{E}\\ Y_{E}\\ Z_{E} \end{array}\right). \end{array}$$

The POS system of tilting photogrammetry technology obtains attitude and position parameters, carries out calibration and naturalization in the calibration field, and naturalizes the center to the center of the camera. The relative angle element and relative line element of tilting camera and downward-looking camera can be obtained. According to the relative relationship, the position and attitude result of the POS system can be decomposed to each sub-camera, and then the external orientation element of the tilting image can be obtained. Since the tilted image has a certain tilt angle, the same method cannot be used to restore the position relation of the tilted image as the conventional image. However, since the photographic center and the image point of the tilted image are still in a straight line, the collinear equation is satisfied, as shown in the formula below:

(5) $$\begin{array}{c} \left[\begin{array}{c} X_{A}-X_{S}\\ Y_{A}-Y_{S}\\ Z_{A}-Z_{S} \end{array}\right]=\lambda \left[\begin{array}{ccc} a_{1} & a_{2} & a_{3}\\ b_{1} & b_{2} & b_{3}\\ c_{1} & c_{2} & c_{3} \end{array}\right]\left[\begin{array}{c} x\\ y\\ -f \end{array}\right]. \end{array}$$

Expand formula (5) to get three equations and divide the first and second equations by the third formula, respectively, as shown in the formula below:

(6) $$\begin{array}{c} \left\{\begin{array}{c} X_{A}-X_{S}=Z_{A}-Z_{S}\frac{a_{1}x+a_{2}y-a_{3}f}{c_{1}x+c_{2}y-c_{3}f}\\ Y_{A}-Y_{S}=Z_{A}-Z_{S}\frac{b_{1}x+b_{x}y-b_{3}f}{c_{1}x+c_{2}y-c_{3}f} \end{array}\right.. \end{array}$$

After the common factors are removed and the coefficients in formula (6) are expressed with new symbols, the simplification is shown in the formula below:

(7) $$\begin{array}{c} \left\{\begin{array}{c} X=\frac{a_{11}x+a_{12}y-a_{13}}{c_{31}x+c_{32}y+1}\\ Y=\frac{b_{21}x+b_{22}y-b_{23}}{c_{31}x+c_{32}y+1} \end{array}\right.. \end{array}$$

The above equation is the central projection configuration equation when the ground is approximately horizontal, also known as the perspective transformation formula, which represents the transformation relationship between two corresponding points on the plane. According to the spatial position and attitude of the image obtained from POS data, combining the above three formulas and fixing the size of ZA, the four corners of the inclined image (including the down-view image) can be projected onto the same elevation plane. Many irregular polygons can be obtained on this elevation plane, and the overlapping relationship between images can be judged. The process of automatic matching of multi-view images is the process of connecting points and constructing a network. The connection point network must optimize the following four types of parameters: POS (GPS/IMU) observation error of class A; The position deviation between class B camera lens and GPS/IMU platform; Related parameters of class C camera; and Class *D* flight attitude parameters. Different types of parameters have corresponding optimization modes in the adjustment calculation, so a configuration file is needed to control the optimization modes of different parameters in the calculation. Therefore, configuration files (group files) need to be made before optimization, as shown in Table 1.

The article "Application of Realistic 3D Model in Building Prefabricated Nanomaterial Structure" was retracted in 2023. Reasons: signs of a paper mill; suspected computer-generated content; unreliable results or conclusions; concerns about the data.

The image control points are inserted into the constructed area network, and the control points laid out are individually adjusted for testing. On the premise of ensuring the accuracy of control points, all connection points are combined to realize the overall area network adjustment, and the whole area network is naturalized to the projection coordinate system defined by the project. If the accuracy of pixel points does not meet the requirements, the automatic filtering and manual interpolation of regional network adjustment are repeated until the accuracy meets the requirements. At the end, a regional network with strong stability and high accuracy is constructed. Every object in real life has its surface details, namely, various textures. Surface texture can usually be divided into color texture and geometric texture. The color texture is the use of color or shade changes to show the surface details of the object; geometric texture, caused by irregular small concave and convex, is a surface texture based on the microscopic geometry of an object's surface. For the definition of texture, there are discrete method, continuous function method, parameter method, and other definition methods. The texture function below can simulate coarse cloth texture as shown in the formula below:

(8) $$\begin{array}{c} f\left(u,v\right)=A\left(\cos\left(pu\right)+\cos\left(qv\right)\right). \end{array}$$

The texture model can be defined by parameters, which can be described in the textual text, especially for defining different texture models for each scene composed of a scene. When the texture is used, it is explained and mapped by a general program, so it can also be called procedural texture definition. In order to map 2D texture to the 3D object surface, it is necessary to create object space coordinates (*x*, *y*, *z*). The correspondence to the texture space (*u*, *v*) corresponds to parameterization of object surfaces. For parametric surfaces, the correspondence is readily available. For example, a cylinder *x*^2^+ *y*^2^ = 1(0≤*z* ≤ 1) can be written as shown in the formula below:

(9) $$\begin{array}{c} \left\{\begin{array}{c} x=\cos\left(2\Pi u\right)\\ y=\sin\left(2\Pi u\right)\\ z=v \end{array}\right.. \end{array}$$

0 ≤ *u* ≤ 1, 0 ≤ *v* ≤ 1, its inverse formula is shown in the formula below:

(10) $$\begin{array}{c} \left(u,v\right)=\left\{\begin{array}{c} \left(y,z\right)\\ \left(x,z\right)\\ \left(\sqrt{x^{2}+y^{2}}-\frac{z}{x,z}\right) \end{array}\right.. \end{array}$$

Texture mapping requires an appropriate mapping transformation for planar polygons or defined surfaces, if the scene space parameters are too sparse, that is, Δ*u*, Δ*v*_is_ too large, then all points mapped to the display screen are scattered, and continuous real area images cannot be formed. On the contrary, if Δ*u*, Δ*v* is too small, the multi-point on the surface will be mapped to a point on the screen, and the display speed will be slow.

The article "Application of Realistic 3D Model in Building Prefabricated Nanomaterial Structure" was retracted in 2023. Reasons: signs of a paper mill; suspected computer-generated content; unreliable results or conclusions; concerns about the data.

## 4. Experiments and Analysis

All the operations of assembling concrete structural components are based on the structural models imported into Revit by WinC software. The method of data sharing of structural model and model sharing avoids repeated modeling in the stage of in-depth design of the assembled concrete structure, which fully meets the requirements of the forward design of BIM technology. At the present stage, the structural design principle of prefabricated concrete building and cast-in-place concrete building in China is the same, that is, it is equivalent to a cast-in-place concrete building. However, in practical application, designers will seek according to relevant specifications and take corresponding measures to ensure that the prefabricated concrete building achieves the same effect as a cast-in-place concrete building. At the present stage, the structural design of prefabricated buildings is based on the traditional cast-in-place concrete structure design, but there are many differences between the two in actual engineering design, such as the design range, design accuracy, number of structural drawings, and pattern expression [18]. On the basis of cast-in-situ concrete structure design, there are more than two contents: precast component splitting design and precast component deepening design. The separation of prefabricated buildings is the basis of the whole prefabricated structure design. The factors affecting the separation design of prefabricated buildings include the rationality of the structure of building functional nanomaterials, the feasibility and convenience of production, transportation, and installation. The resolution of prefabricated concrete structure engineering includes: determining the boundary between cast-in-place and prefabricated; determine where the structural components are split; determine the relationship between the post-pouring area and the prefabricated components, including the relationship between the relevant prefabricated components. For example, the floor is determined to be laminated plate, because the steel bar of the laminated plate needs to be extended to the support for anchorage, the support beam must also have a laminated layer accordingly; determine the separation location between components, such as column beam wallboard members at the joint. From the point of view of the structure, the structure should be divided into the rationality of the structure, such as the composite floor supported by four sides, the direction of plate splitting (plate seam) should be perpendicular to the long side; the joint of the component is selected in the part of low stress; and the sleeve joint of column-beam structure system of high-rise building should avoid plastic hinge position. Specifically, the end of the top beam of the column foot of the first layer and the tension side column of the column beam structure should not be designed for sleeve connection [19, 20]. Avoid the plastic hinge position of the beam end, and the connecting node of the beam should not be located within the range of H from the beam end; unify and reduce component specifications as much as possible; it should be coordinated with the separation of adjacent related components, such as the separation of composite plates and support beams [21]. Texture mapping, through a certain mapping function, the texture of the two-dimensional space is mapped to the surface of the three-dimensional object is essentially a coordinate system to a coordinate system transformation. Texture mapping, usually have forward mapping and reverse mapping forward mapping, is in the texture space, defines a two-dimensional texture function, through the mapping of two-dimensional texture to three-dimensional object surface, and then projection transformation, projection to the image space. Reverse mapping is a process from screen space to texture space. Reverse mapping, which accesses pixels of screen space in a sequential manner, obtains coordinate information, and assigns values to tilted textures on pixels, is a forward mapping process. Through the orientation of the inclined image, the external orientation elements of the inclined image can be calculated, combined with the external orientation elements of the inclined aerial film, and the texture of the inclined image can be mapped to the white model of the building. The process of tilted texture mapping usually includes: the selection of the optimal image containing all tilted images of the house surface, the judgment of the occlusion of the house surface, and the correction and editing of the mapped texture to complete the automatic mapping of a tilted texture, as shown in Figure 4.

The article "Application of Realistic 3D Model in Building Prefabricated Nanomaterial Structure" was retracted in 2023. Reasons: signs of a paper mill; suspected computer-generated content; unreliable results or conclusions; concerns about the data.

Dji's Altizure ground console is a multi-platform application that can be used not only on Android and ios mobile devices, but also on Windows PCS. The software itself does not support remote data transmission, so the flight data must be extracted by relying on the memory card equipped with the airborne camera of the UAV, and the flight altitude of the extracted UAV aerial photography data should be manually classified, recorded and saved. The flight altitude recorded in the flight process is shown in Table 2.

In the process of building a 3D real-scene model with ContextCapture series software on the Bentley platform, the geometric dimensions of model space are measured, and the actual precision and model precision of 3D real scene model are extracted. The experimental results show that the modeling method based on airborne LiDAR and tilt photography achieves good results in the construction of urban building models. This modeling method can successfully build the model of the building in the experimental area, with high modeling efficiency, and the established urban building model has high precision and good real-scene effect. The precision of the building model meets the requirements of 1 : 1000 mapping, with measurable accuracy, and elevation accuracy is better than 30 cm. Experimental results show that this modeling method is feasible and advanced and improves the working efficiency and quality of the existing modeling method. In the assembled concrete shear wall structure, there are some differences in the disassembling methods of connecting beam and frame beam [22]. Even beam and frame beam are above the damage form and stress analysis calculation, coupling beam, and frame beam split method are different. Even the beam is mainly shear stress form, and even the beam is mainly connected to shear walls, so in the design of split, even the beam can be split separately, and coupling beam can also be a common split shear wall as a whole. Frame beam is divided into a main beam and secondary beam, generally the span of the main beam is large, if the main beam and secondary beam as a whole to split, will increase the production difficulty of prefabricated components factory, at the same time, it is easy to damage the primary and secondary beam nodes in transportation, will also bring great inconvenience to the lifting and installation, so the main beam and secondary beam generally separate split [23]. The joint parts of the primary and secondary beams are split, and the joint parts are further designed to ensure that the components produced after splitting can be accurately installed on the construction site. In the prefabricated structure, the column is generally divided according to the height of the floor. According to The Relevant Provisions of the Technical Specification of Prefabricated Prestressed Concrete Integrated Frame JGJ224-2010, the column can be divided into multiple columns. However, due to the multi-section column in demolding, there is a lot of inconvenience in the process of transportation and hoisting, and in the process of transportation and installation, it is easy to damage the steel connection part, resulting in the deformation of the joint steel, which will cause the perpendicularity of the component is difficult to control. Therefore, in the actual separation, often according to the height of separation for a single column, in order to control the verticality of components, simplify demoloming transportation and lifting difficulty, ensure that components to. And assembly type structure overall quality safety. The size of floor components can be divided into one-way floor and two-way floor, for the resolution of floor components can be divided into all one-way floor or one-way floor and two-way floor mixed assembly form. There are different modes of stress and failure characteristics between one-way plate members and two-way plate members. If the combination of single and double plate members is used to split, the connection between the two is realized through the interaction of overlapping layer and distributed steel bars. At this time, the mode of stress in the plate will adversely affect the one-way plate. Prefabricated composite floor slabs are commonly used in floor components of prefabricated residential buildings. Considering the hoisting and transportation process of prefabricated components, their size should be controlled [24, 25]. To facilitate truck transportation, the width of the prefabricated floor plate is generally not more than 3 m, and the span is generally not more than 5 m. In a room, the precast bottom plate should be as wide as possible to choose split, in order to reduce the type of precast bottom plate when the span of the floor is not large, the plate joint can be set in the part of the internal partition, the template joint after the completion of the construction of the internal partition cannot be processed. The separation of the precast floor also needs to consider the lighting position of the room, generally speaking, the plate joint should avoid the lighting position of the toilet strong and weak electric pipeline intensive floor slab is generally used in the way of the cast-in-place concrete floor slab. When designing the precast members in detail, it is necessary to calculate and design the position of the embedded parts [26]. Embedded parts mainly include hoisting embedded parts, demolded embedded parts, and inclined support embedded parts, these three embedded parts can be designed according to the situation for common embedded parts such as wall panel demolded embedded parts and inclined support embedded parts can be designed for common, not only can reduce the workload can also reduce the cost. The position of the embedded parts can be selected according to the principle of the minimum bending moment when hoisting and demolding the precast members with equal sections. For hoisting embedded parts, when the maximum positive bending moment and the maximum negative bending moment produced under the action of dead weight are equal, the absolute value of bending moment endured by the whole precast member is minimum. For demolded embedded parts, it will be affected by the joint action of dead weight and bond force (between the precast member and the die), but the bond force can be considered as uniform distribution, so the position of the embedded parts determined when the absolute bending moment of the precast member is minimum is the same as that determined when only considering the gravity effect. Compared with cast-in-place concrete, prefabricated concrete buildings are divided into two parts, namely, precast component splitting and component deepening design [27, 28]. The required structural model is directly imported and obtained by the structural calculation software of WinC, avoiding repeated modeling, while the prefabricated components (prefabricated beams, prefabricated columns, and prefabricated panels) are split and designed. Check the hoisting load of the embedded parts in the deepening design of the precast composite beam precast column precast composite beam and other components, especially for the reinforcement component connection node embedded parts and other parts of the deepening design. Use Revit software to produce 3D drawings directly, which is also the most important part of the in-depth design : Instead of CAD drawing, it avoids repeating drawing and reduces the workload of engineers. Meanwhile, 3D deepening drawing is more conducive to later construction and operation and maintenance.

The article "Application of Realistic 3D Model in Building Prefabricated Nanomaterial Structure" was retracted in 2023. Reasons: signs of a paper mill; suspected computer-generated content; unreliable results or conclusions; concerns about the data.

## 5. Conclusion

In this paper, based on BIM technology to build 3D real model method, combined with UAV image data acquisition technology, aiming at the influence factors of UAV tilt image data acquisition model accuracy of the optimal way, the application of 3D real model in road and bridge engineering is studied. Based on the reconstruction theory of 3D real scene model, the influence of single shot multiple data acquisition and single shot multiple data acquisition on model error of UAV oblique photography was compared and analyzed. Combined with the principle of UAV aerial photography, the factors influencing the accuracy of 3D real scene model are comprehensively studied. In the process of UAV oblique photography, the heading overlap rate of flight height and the side overlap rate of camera tilt Angle are selected as the influencing factors of model accuracy. Through the modeling experiments of an actual badminton court under different influencing factors, the precision errors of the model, and the actual court are compared and analyzed, and an effective model precision control method is obtained; The BIM-based 3D real-scene modeling method is adopted in combination with UAV tilt photography data acquisition technology, and the application research of BIM-based 3D real scene model is carried out for project management and bridge appearance inspection in road and bridge engineering.

## Figures and Tables

**Figure 1:** Application of 3D model in building assembly structure.

**Figure 2:** Modeling procedure.

**Figure 3:** Schematic diagram of collinear equations.

**Figure 4:** Tilt texture automatic mapping process.

**Table 1:** Parameter optimization.

Parameter type	The optimized model
A	The corresponding parameters of each image involved in the calculation were optimized separately and did not affect each other
B	Images taken by the same camera should have the same optimization value (fixed camera position)
C	Images taken by the same camera should have the same optimization value (camera lens remains unchanged)
D	The optimization values of the images taken by the same camera and the same route should be consistent

The article "Application of Realistic 3D Model in Building Prefabricated Nanomaterial Structure" was retracted in 2023. Reasons: signs of a paper mill; suspected computer-generated content; unreliable results or conclusions; concerns about the data.

**Table 2:** The recorded altitude of five flights.

Flight number	The first time	The second time	The third time	The fourth time	The fifth time
Flight height (m)	60	80	100	120	140

## Data Availability

The data used to support the findings of this study are available from the corresponding author upon request.
